# MicroRNA-17-5p Protects against Propofol Anesthesia-Induced Neurotoxicity and Autophagy Impairment via Targeting BCL2L11

**DOI:** 10.1155/2022/6018037

**Published:** 2022-06-28

**Authors:** Mingyu Xiu, Hengfei Luan, Xiaojiao Gu, Chuang Liu, Deming Xu

**Affiliations:** Department of Anesthesiology, The First People's Hospital of Lianyungang, Lianyungang 222000, China

## Abstract

**Background:**

Propofol (PPF) has been shown in studies to cause cognitive impairment and neuronal cell death in developing animals. PPF has been demonstrated to decrease the expression of microRNA-17-5p (miR-17-5p) in a recent study. Nonetheless, the function of miR-17-5p in PPF-induced neurotoxicity and related mechanisms is uncharacterized.

**Methods:**

After the induction of neurotoxicity by treating the SH-SY5Y cells with PPF, qRT-PCR was conducted to evaluate the level of miR-17-5p. Using MTT and flow cytometry, cell viability and apoptosis rate were assessed, respectively. Interaction between miR-17-5p and BCL2 like 11 was (BCL2L11) studied using a Luciferase reporter assay. With the help of western blot analysis, we determined the level of proteins of apoptosis-related genes and autophagy-related markers.

**Results:**

In SH-SY5Y cells, PPF treatment induced neurotoxicity and downregulated miR-17-5p expression. In SH-SY5Y cells post-PPF exposure, overexpression of miR-17-5p increased cell viability and decreased apoptosis. Consistently, miR-17-5p mimics mitigated PPF-generated autophagy via inhibition of Atg5, Beclin1, and LC3II/I level and elevation of p62 protein expression. In addition, BCL2L11, which was highly expressed in PPF-treated SH-SY5Y cells, was directly targeted by miR-17-5p. Further, in PPF-treated SH-SY5Y cells, overexpressed BCL2L11 counteracted the suppressing behavior of miR-17-5p elevation on PPF-induced apoptosis.

**Conclusion:**

Overexpressed miR-17-5p alleviates PPF exposure-induced neurotoxicity and autophagy in SH-SY5Y cells via binding to BCL2L11, suggesting the possibility that miR-17-5p can serve as a candidate in the treatment of neurotoxicity (caused by PPF).

## 1. Introduction

Ever-increasing evidence reveals that different kinds of anesthetics can lead to long-term cognitive dysfunction and adverse effects on the development of neurons [1]. In addition, anesthesia often causes developmental neurotoxicity such as neurodegeneration, neurogenetic change, synaptogenesis, and brain circuit damage [2]. Based on the rapid onset and minimal negative postoperative effects, PPF is widely used to induce and maintain sedation as well as anesthesia [3]. PPF is still an anesthetic that should be used with caution in most clinical paediatric settings since it always causes bradycardia, heart failure, metabolic acidosis, and other complications [4, 5]. In developing mice, even subanesthetic doses of PPF can cause cell death, aberrant dendrite formation, and cognitive impairment, according to documents [6, 7]. All these effects raise concerns about the safety of PPF in paediatric anesthesia. Clinical studies have attributed neurotoxicity and neurogenic injury to PPF [8, 9]. The complex mechanisms of neurotoxicity induced by PPF include intracellular calcium dysregulation, mitochondrial division, neuroinflammation, and abnormal neurotrophic protein expression [10–12]. Recent research has revealed that the mechanisms underlying PPF may exert a role in the establishment of novel effective therapeutic methods to avoid neurotoxicity in the underdevelopment brain [13]. Therefore, biological biomarkers must be investigated in order to prevent and treat neurotoxicity caused by PPF exposure.

miRNAs, which are endogenous noncoding RNA molecules with lengths ranging from 18 to 25 nucleotides, can regulate various biological processes via targeting and regulating the downstream messenger RNAs (mRNAs) expression at the posttranscriptional level [14–16]. Plenty of studies have identified the influence of miRNAs in the modulation of neurotoxicity mediated by PPF. For example, miR-582-5p mitigates PPF-generated neuron apoptosis by inhibition of ROCK1 in newborn rats [17]. PPF anesthesia reduces the expression of miR-132 and decreases the number of dendritic spines in the hippocampus [18]. miR-141-3p knockdown alleviates PPF-mediated inhibition on neural stem cell neurogenesis by targeting IGF2BP2 [19]. As previously reported, miRNAs also participate in the process of PPF-mediated autophagy. Downregulated endogenous expression of miR-20b weakens the protective role of PPF and causes accentuation on autophagy [20]. Interestingly, miR-17-5p has been validated to bind with STAT3 and thus regulating the growth of cortical neuron neurite [21]. In addition, miR-17-5p, which displays low level after PPF treatment, is involved in cardiomyocyte apoptosis induced by ischemia/reperfusion (I/R) [22]. Though, the biological functionality, as well as molecular mechanisms of miR-17-5p in PPF-induced neurotoxicity, has not been evaluated.

BCL2-like 11 (BCL2L11), a member of the Bcl-2 family, is found on chromosome 2q12-q13. BCL2L11 is anticipated to share a binding site with miR-17-5p, according to bioinformatics analysis. The human BCL2L11 gene comprises important death-decision makers in the process of apoptosis [23]. BCL2L11 abrogates miR-92a-induced suppression on cell apoptosis and caspase-3/7 activity [24]. Nonetheless, the BCL2L11 role in PPF-induced neurotoxicity remains unclear.

In our current investigation, what we intended to decipher is the functionality of miR-17-5p in regulating PPF-treated SH-SY5Y cell apoptosis and autophagy and the underlying mechanisms associated with miR-17-5p. The current study may explore a new candidate target for treating neurotoxicity (caused by PPF exposure).

The paper's organization paragraph is as follows: the materials and methods are presented in Section 2.  Section 3 discusses the experiments and results. Finally, in Section 4, the research work is concluded with discussion.

## 2. Materials and Methods

### 2.1. Cell Culture

We purchased the human neuroblastoma SH-SY5Y cell line from China Center for Type Culture Collection (CCTCC) and plated in 96-well plates (BD Biosciences, USA) and incubated in DMEM (Invitrogen, USA) containing FBS (10%) (Invitrogen) and penicillin (100 U/mL) (LianShuo, Shanghai, China) under humid conditions with 5% CO_2_ at 37°C. 1, 5, 10, and 20 *μ*g/ml PPF (2,6-diisopropylphenol, Merck & Co., USA) were utilized for the overnight treatment of SH-SY5Y cells, and phosphate buffer was used as a blank control.

### 2.2. Cell Transfection

RiboBio (Guangzhou, China) provided the miR-17-5p mimics and negative control (NC) used for the overexpression of miR-17-5p and as the control, respectively. pcDNA3.1/BCL2L11 was used to increase BCL2L11 expression, with an empty vector pcDNA3.1 (GenePharma). We transfected the miR-17-5p and NC mimics (50 nM each) pcDNA3.1/BCL2L11 (10 nM) or empty pcDNA3.1 (10 nM) in SH-SY5Y cells with Lipofectamine 2000 for 48 h. The cells transfected by Lipofectamine 2000 with scrambled sequences served as NC.

### 2.3. 3-(4,5-Dimethylthiazol-2-yl)-2,5-Diphenyltetrazolium Bromide (MTT) Assay

With the help of the MTT assay, we performed the identification of SH-SY5Y cell viability as instructed by the supplier. In 96-well plates, the SH-SY5Y (5 × 10^4^ cells/well) cells were seeded. After cell transfection, the cell viability with or without PPF treatment was detected using a MTT kit (Promega, USA), followed by adding the solution of MTT (20 *μ*l, 0.5 mg/ml) into each well for continuous cell culturation for 4 h. Formazan crystals were dissolved by carefully removing the medium, adding 100 *μ* L dimethyl sulfoxide and incubating the cells at 37°C for 10 min. Through a microplate reader (Thermo Fisher Scientific), the O.D. was achieved at 570 nm.

### 2.4. Isolation of RNA and qRT-PCR Evaluations

The Ultra HiFidelity PCR Kit (Tiangen) was utilized for total RNA extraction. RNA concentrations were quantified by Nanodrop (Thermo Fisher Scientific, USA). We adopted the TaqMan miRNA reverse transcription kit (Beyotime) to reverse transcribe RNA (total of 1 *μ*g) to cDNA. The qRT-PCR was then conducted via SYBR Green (Takara, Dalian, China) on Applied Biosystems (Thermo Fisher Scientific). Detailed conditions were that 10 min at 95°C, and 40 cycles at 95°C for 10 sec and at 60°C for 30 sec (for MIDN, MYLIP, BCL2L11 and glyceraldehyde-3-phosphate dehydrogenase (GAPDH)), 10 min at 95°C, and 40 cycles at 95°C for 10 sec and 2 at 60°C and 1 min at 95°C, 30 sec at 55°C, and 30 sec at 95°C (for miR-17-5p). Calculation for the relative gene expression was achieved via 2^-*ΔΔ*Ct^ method [25]. U6 and GAPDH were, respectively, utilized as the internal references for miR-17-5p and BCL2L11. The study includes the underlined primer sequences: miR-17-5p forward: 5′-CCGGGTCAGAATAATGTCAAAGTGCTTACAGTGCAGGTAGTGATATGTGCATCTACTGCAGTGAAGGCACTTGTAGCATTATGGTGACTTTTTG-3′, reverse: 5′-AATTCAAAAAGTCACCATAATGCTACAAGTGCCTTCACTGCAGTAGATGCACATATCACTACCTGCACTGTAAGCACTTTGACATTATTCTGAC-3′; BCL2L11 forward: 5′-CAAGGAGGATGCCTCTTCC-3′, reverse: 5′-CTTCCTGAGACCTGCTGTC-3′; GAPDH forward, 5′-CCTCCTGTTCGACAGTCAG-3′, reverse: 5′-CATACGACTGCAAAGACCC-3′; U6 forward: 5′-CTTTGGCAGCACATATACCA-3′, reverse: 5′-CTCATTCAGAGGCCATGCT-3′.

### 2.5. Flow Cytometry (FC) Analysis

With the help of the Annexin V-FITC Apoptosis Detection Kit (Vazyme, Nanjing, China), we analyzed the SH-SY5Y cell apoptosis. The cells were centrifuged and resuspended in binding buffer after being treated with PPF (100 *μ*l) (MultiSciences, Hangzhou, China). Then, we added the Annexin V-FITC and PI (5 *μ*l each) reagents into the cells for culturation for 15 min with light. Analyzation of cell apoptosis was achieved using FACS flow cytometer (Attune, Life Technologies, Germany).

### 2.6. Western Blot (WB) Analysis

After PBS washing, the centrifugation (at 10,000 × g) of lysed cells was carried out for 10 min at 4°C. A Bradford Protein Assay kit (Invitrogen, USA) was adopted for the determination of total protein concentrations. We separated the protein samples (25 *μ*g) by SDS-PAGE (10%), followed by transferring them onto PVDF membranes (Standards, Shanghai, China) that were subsequently sealed with skimmed milk (5%) at 37°C for 1.5 h. Incubation of the membranes was performed with primary antibodies against Bcl-2 (1 : 1000 dilution, ab32124, Abcam), Bax (1 : 5000 dilution, ab32503, Abcam), Cleaved-caspase-3 (1 : 500 dilution, ab32042, Abcam), Atg5 (1 : 5000 dilution, ab108327, Abcam), Beclin 1 (1 : 2000 dilution, ab207612, Abcam), LC3 (0.5 --2 *μ*g/ml, ab48394, Abcam), p62 (1 : 10000 dilution, ab109012, Abcam), BCL2L11 (1 : 1000 dilution, ab32158, Abcam), and GAPDH (1 : 2500 dilution, ab9485, Abcam) for 24 hrs at 4°C. After that, the membrane was incubated with the secondary antibody at 37°C for 2 h. An enhanced chemiluminescence kit (Takara, Dalian, China) and ImageJ software [26] were, respectively, utilized for signal visualization and blot analyzation.

### 2.7. Dual-Luciferase Reporter (DLR) Assay

DNA sequencing was used for confirming the wild type (WT) and mutant (Mut) 3′-UTR sequences of BCL2L11. The BCL2L11-WT and BCL2L11-Mut vectors were constructed by amplifying and inserting the WT and Mut 3′-UTR sequences of BCL2L11 into the luciferase reporter pmirGLO (Promega, USA). In 96 well-plates, SH-SY5Y cells were plated and grown for 24 h at 37°C. After removing the culture medium, Lipofectamine 2000 was adopted for cotransfection of BCL2L11-WT or BCL2L11-Mut vectors with mimics (miR-17-5p or NC) in SH-SY5Y cells. Post 48 h of transfection, we used a DLR Assay Kit (Promega, USA) to determine the relative luciferase activity (LA) of BCL2L11-WT and BCL2L11-Mut vectors with Renilla LA as normalization.

### 2.8. Statistical Analysis

Each analysis was done three times, and the results were expressed as mean standard deviation. In order to perform the statistical analysis, we used GraphPad Prism 6.0 (USA). The one-way ANOVA or Student's *t* test, followed by Tukey's post hoc test, was utilized to analyze variations between two or more groups. Less than a 0.05 *p* value indicates statistical significance.

## 3. Results

### 3.1. PPF Treatment Induces Neurotoxicity in SH-SY5Y Cells and Downregulated miR-17-5p Expression

For investigating the impact of neurotoxicity caused by anesthesia, SH-SY5Y cells were exposed to PPF or phosphate buffer treatment (1, 5, 10, or 20 *μ*g/ml), followed by in vitro evaluation of their cell viability. MTT assay illuminated that compared with the cells treated with phosphate buffer, and the viability of the SH-SY5Y cells was inhibited by 5, 10, and 20 *μ*g/ml of PPF, suggesting that PPF treatment resulted in neurotoxicity in SH-SY5Y cells (Figure 1(a)). The miR-17-5p level was further tested by qRT-PCR. The results of qRT-PCR revealed a dose-dependent lower trend in miR-17-5p concentrations in SH-SY5Y cells (exposed to PPF) relative to the control (Figure 1(b)). Because the SH-SY5Y cell's viability was approximately 50% at 10 *μ*g/ml of PPF, PPF at a 10 *μ*g/ml dose was selected for subsequent cellular experiments. The viability of SH-SY5Y cells was then tested at 0, 6, 12, 24, and 48 h. As a result, SH-SY5Y cell viability was reduced at 12, 24, and 48 h when compared to the NC group (Figure 1(c)). Consistently, the expression level of miR-17-5p was also downregulated with the increase of time after 10 *μ*g/ml of PPF treatment (Figure 1(d)). There was a dose and time-dependent decrease in miR-17-5p expression following PPF treatment of SH-SY5Y cells, as demonstrated by the above results.

### 3.2. miR-17-5p Alleviates PPF-Induced SH-SY5Y Cell Injury

Subsequently, miR-17-5p mimic transfection was carried out with the aim of probing into the effect of the miR-17-5p upregulation on PPF-injured SH-SY5Y cells. Notably, significantly elevated expression of miR-17-5p was indicated in SH-SY5Y cells (exposed to PPF) after miR-17-5p mimic transfection than with the transfection of NC mimics (Figure 2(a)). For the assessment of the fact that whether miR-17-5p exerts the regulatory function in PPF-induced neurotoxicity, MTT assay was conducted. The observed results indicated the elevation of miR-17-5p significantly rescued PPF-injured cell viability (Figure 2(b)). In addition, the apoptosis of SH-SY5Y cells was investigated by FC and WB analysis, which demonstrated that PPF treatment significantly increased cell apoptosis rate as compared to the Con + NC mimic group. Overexpressed miR-17-5p was responsible for increased apoptosis in PPF-treated cells (Figures 2(c) and 2(d)). The protein levels of the markers associated with apoptosis (Bax and Cleaved-caspase-3) were downregulated after PPF treatment, but the reduced levels were reversed with the miR-17-5p mimic transfection. In contrast, overexpressed miR-17-5p partially abrogated the promoting impact of PPF-treatment on the protein levels of Bax, a marker associated with apoptosis (Figure 2(e)). Conclusively, overexpressed miR-17-5p mitigated PPF-injured SH-SY5Y cells and inhibited PPF-induced neuron apoptosis.

### 3.3. miR-17-5p Inhibits PPF-Induced Autophagy in SH-SY5Y

Previous research has identified that miR-17-5p possesses antiautophagy effect in human diseases [27, 28]. Therefore, we examined the protein levels of markers related to autophagy (Atg5, Beclin1, p62, and LC3) in SH-SY5Y cells. Specifically, Beclin1 serves as a marker for autophagy. LC3II/I and p62 are markers of early and late autophagy, accordingly. When compared to the Con + NC mimic group, aberrant autophagy was seen in the propofol + NC mimic group, including enhanced levels of autophagy of Atg5, Beclin1, and LC3II/I ratios and decreased level of p62 protein. Interestingly, comparing with the propofol + NC mimic group, transfecting miR-124 mimics significantly reduced the protein levels of Atg5, Beclin-1, and LC3II/I ratios and restored p62 protein levels (Figures 3(a)–3(e)). These findings elaborated the implication of miR-17-5p in the suppression of autophagy.

### 3.4. miR-17-5p Targets BCL2L11 in SH-SY5Y

To probe into the underlying mechanism through which miR-17-5p alleviates PPF-induced neurotoxicity, prediction of downstream targets of miR-17-5p was carried out via starBase online website (https://starbase.sysu.edu.cn/) with the screening condition of AgoExpNum > 60. The predicted results manifested that miR-17-5p shares 3′-UTR binding sites with MIDN, MYLIP, and BCL2L11. By performing qRT-PCR, the levels of MIDN, MYLIP, and BCL2L11 mRNA expression in SH-SY5Y cells were assessed, and only BCL2L11 level was decreased in SH-SY5Y cells after miR-17-5p mimic transfection relative to the NC mimic-transfected cells (Figure 4(a)). WB analysis was used to examine the amounts of BCL2L11 protein in SH-SY5Y cells. Upregulation of miR-17-5p dramatically reduced BCL2L11 protein levels, according to the findings (Figures 4(b) and 4(c)). An LR assay was conducted in order to validate that the 3′-UTR sequence of BCL2L11 is specifically targeted by miR-17-5p. Predicted pairing target region of BCL2L11 and miR-17-5p was presented in Figure 4(d). It was found that compared to luciferase activity (LA) in cells cotransfected with NC mimics and BCL2L11-WT, the LA was inhibited significantly after being cotransfected with miR-17-5p mimics and WT BCL2L11 3′-UTR; however, luciferase activity was not significantly changed in cells cotransfected with Mut BCL2L11 3′-UTR and miR-17-5p mimics or NC mimics (Figure 4(e)). Subsequent qRT-PCR and WB analyses exhibited an elevated level of BCL2L11 at both transcriptional and translational levels after treatment with PPF (Figures 4(f) and 4(g)). All these experiments illuminated that miR-17-5p bound with BCL2L11 in SH-SY5Y cells and PPF induced the elevation of BCL2L11 expression.

### 3.5. miR-17-5p Targets BCL2L11 to Regulate SH-SY5Y Cell Viability and Apoptosis

To further explore whether miR-17-5p modulates cell viability and apoptosis via targeting BCL2L11, we conducted several rescue experiments using SH-SY5Y cells. qRT-PCR illuminated that BCL2L11 expression was elevated by transfecting pcDNA3.1/BCL2L11 (Figure 5(a)). Similar results were observed in WB analysis that BCL2L11 protein level was increased after pcDNA3.1/BCL2L11 transfection (Figure 5(b)). MTT assay indicated the enhanced level of miR-17-5p exerts the promotive impact on the viability of the SH-SY5Y cells, but this effect was countered after transfection of pcDNA3.1/BCL2L11 (Figure 5(c)). BCL2L11 overexpression counteracted the inhibitory effect of overexpressed miR-17-5p on cell apoptosis, according to FC analysis (Figure 5(d)). Furthermore, WB analysis revealed that increased BCL2L11 partially reversed the miR-17-5p-mediated reduction of Bax and Cleaved-caspase-3 protein levels. In contrast, overexpressed BCL2L11 offsets miR-17-5p elevation-induced promotion on Bcl-2 protein level (Figure 5(e)). Thus, miR-17-5p exerted a protective role in SH-SY5Y cells by downregulating BCL2L11.

## 4. Discussion

Recently conducted preclinical and clinical studies revealed that neonatal prolonged or repeated exposure to anesthesia leads to the increased risk for acute neurotoxicity and long-term cognitive impairment [29]. There is currently no effective way to prevent anesthesia-induced neurotoxicity and cognitive impairments [29]. However, because the use of anesthetics is inevitable in many paediatric procedures, researching techniques to decrease neurotoxicity induced by anesthetics is critical. It has been revealed by previous research that SH-SY5Y human neuroblastoma cells are sensitive to anesthetic-induced neurotoxicity [30]. Hence, SH-SY5Y cells were selected to conduct *in vitro* experiments. PPF, as an effective inducer of nerve injury, can bring about neuron apoptosis and autophagy [31]. Clinical studies also revealed the neuroprotective effects of PPF that PPF treatment protects against I/R or hypoxic injury [32, 33]. In our exploration, the PPF effect on SH-SY5Y cells was first determined by MTT assay, FC, and WS analysis. Findings demonstrated that PPF dose- and time-dependently suppressed the viability of the SH-SY5Y cells. The results are consistent with a recent report showing the inhibition of SH-SY5Y cell viability with the increased PPF concentration [34]. Additionally, after PPF treatment, cell apoptosis rate and autophagy were significantly elevated. Our results verified that PPF treatment induced obvious neurotoxicity in SH-SY5Y cells.

Previous documents have illuminated that miRNAs showed expression levels in the nervous system and implicated in the development of neurological diseases [35, 36]. miR-214-5p reduces contents of serum inflammatory factors and alleviates the cognitive impairment by targeting SUZ12 in Alzheimer's disease mice [37]. miR-23b knockdown alleviates ischemic brain injury via elevating the level of nuclear factor erythroid 2-related factor 2 [38]. Upregulation of miR-29a mitigates aluminum-induced injury to primary hippocampal neurons [39]. miR-17-5p expression is downregulated in paraquat-induced neuro-2a cells, and miR-17-5p depletion has a critical role in dopaminergic neurodegeneration induced by paraquat [40, 41]. The level of miR-17-5p in SH-SY5Y cells exposed to various PPF doses was detected, and the results presented the time- and dose-dependent decrease in its expression. The expression of miR175p increased the survival of PPF-treated cells and inhibited the apoptotic and autophagic processes in SH-SY5Y cells treated with PPF. These discoveries reveal that miR-17-5p is able to play a neuroprotective function in neurotoxicity (caused by PPF) by suppression of apoptotic process and autophagy in SH-SY5Y cells.

Plenty of documents have identified that miRNAs possess the ability to target various mRNAs and modulate the expression of genes to repair neuronal damage in neurodegenerative diseases [42]. By using bioinformatics analysis tools, BCL2L11 was predicated as the downstream target of miR-17-5p. Herein, BCL2L11, which presented elevated expression after PPF treatment, was validated to be directly targeted by miR-17-5p in SH-SY5Y cells. BCL2L11 is believed to play the role of apoptosis facilitator in many diseases [43]. For example, inhibition of BCL2L11 reduces neuron apoptosis in Alzheimer's diseases [44]. In addition, overexpression of BCL2L11 eliminates the miR-338-5p protective role against apoptosis of neurons [45]. Consistent with previous research, our results illuminated that in PPF-treated SH-SY5Y cells, overexpression of BCL2L11 reversed the rise in cell survival and the decrease in apoptotic process in context of miR-17-5p overexpression suggesting the potential of miR-17-5p to alleviate PPF exposure-caused the SH-SY5Y cells apoptosis by targeting BCL2L11.

Finally, our research looked at the role of miR-17-5p in PPF-induced apoptosis, autophagy, and the associated mechanism. The results showed that miR-17-5p, by inhibiting BCL2L11, reduced PPF-induced cell damage. Our study innovatively demonstrated that miR-17-5p may serve as a therapeutic target for the treatment of neurotoxicity caused by PPF. Nonetheless, there were few limitations to this study. First, the protective role of miR-17-5p in SH-SY5Y cells (PPF-induced) was just validated by *in vitro* experiments, and *in vivo* studies are required to evaluate whether miR-17-5p exerts protective function in PPF-induced animal models. Second, due to the complexity of molecular mechanisms, the upstream molecules or downstream signaling pathways of the miR-17-5p/BCL2L11 axis still need further exploration.

## Figures and Tables

**Figure 1:** PPF treatment induces neurotoxicity in SH-SY5Y cells and downregulates miR-17-5p expression. (a) MTT assay was conducted to evaluate the survival of SH-SY5Y cells exposed to elevated concentrations (1, 5, 10, or 20 *μ*g/ml) of PPF. (b) The level of miR-17-5p after treatment with elevated concentrations (1, 5, 10, or 20 *μ*g/ml) of PPF by qRT-PCR. (c) The SH-SY5Y cells after treatment with 10 *μ*g/ml of PPF for 0, 6, 12, 24, and 48 h were used for an MTT assay to determine their viability. (d) The miR-17-5p level in SH-SY5Y cell postexposure with 10 *μ*g/ml of PPF at different time points was subjected for qRT-PCR evaluations. ^∗^*p*, ^∗∗^*p*, and ^∗∗∗^*p* values less than 0.05, 0.01, and 0.001, accordingly.

**Figure 2:** Functional experiments focusing on the impact of miR-17-5p on PPF-caused neurotoxicity. (a) By utilizing qRT-PCR, the miR-17-5p transcriptional level was examined in SH-SY5Y cells with or without 10 *μ*g/ml of PPF treatment posttransfection with miR-17-5p or NC mimics. (b) The survival of SH-SY5Y cells was measured via MTT in the groups of Con + NC mimics, Con + miR − 17 − 5p, propofol + NC mimics, and propofol + miR − 17 − 5p. (c, d) FC analysis was conducted to assess the apoptosis process in the abovementioned groups. (e) Representative results of WB showed the translational levels of Bcl-2, Cleaved-caspase-3, and Bax in various groups. ^∗^*p*, ^∗∗^*p*, and ^∗∗∗^*p* values less than 0.05, 0.01, and 0.001, accordingly.

**Figure 3:** miR-17-5p inhibits PPF-induced autophagy in SH-SY5Y. (a)–(e) Protein levels of proteins related to autophagy (Atg5, Beclin1, LC3, and p62) in transfected SH-SY5Y cells with miR-17-5p or NC mimics with or without PPF (10 *μ*g/ml) were measured by WB. ^∗^*p*, ^∗∗^*p*, and ^∗∗∗^*p* values less than 0.05, 0.01, and 0.001, accordingly.

**Figure 4:** BCL2L11 is directly targeted by miR-17-5p in SH-SY5Y. (a) qRT-PCR examined the level of MIND, MYLIP, and BCL2L11 in SH-SY5Y cells with miR-17-5p or NC mimic transfection. (b, c) BCL2L11 protein levels were measured in SH-SY5Y cell posttransfection with miR-17-5p or NC mimics by WB. (d) Predicated binding region between miR-17-5p and BCL2L11 through Targetscan. (e) Validation of the combination between miR-17-5p and BCL2L11 via DLR assay. (f, g) BCL2L11 transcriptional and translational level was tested in SH-SY5Y cells treated with PPF or phosphate buffer by qRT-PCR and WB analysis, respectively. ^∗∗^*p* < 0.01.

**Figure 5:** The influence of miR-17-5p on SH-SY5Y viability and apoptosis via modulating BCL2L11. Postexposure with PPF (10 *μ*g/ml) for 24 h, rescue experiments were conducted. (a, b) Overexpression efficacy of BCL2L11 in SH-SY5Y cells was, respectively, evaluated by qRT-PCR and WB evaluations. (c, d) MTT assay and FC analysis were performed for evaluating SH-SY5Y cell viability and apoptosis after transfection of NC mimics, miR-17-5p mimics, and miR − 17 − 5p mimics + pcDNA3.1/BCL2L11. (e) The translational levels of Bcl-2, Bax, and Cleaved-caspase-3 were estimated by WB in SH-SY5Y cells with plasmids transfection. ^∗^*p*, ^∗∗^*p*, and ^∗∗∗^*p* values less than 0.05, 0.01, and 0.001, accordingly.

## Data Availability

Data will be provided upon request to the authors.
